The article "Application of Outlier Detection Model in Korean Language and Culture Communication System Based on Artificial Intelligence" was retracted in 2023. Reasons: unreliable results or conclusions; concerns about the data; concerns about the peer review; concerns about the citations.

# Application of Outlier Detection Model in Korean Language and Culture Communication System Based on Artificial Intelligence

**DOI:** 10.1155/2022/6414112

**Published:** 2022-10-15

**Authors:** Qiao Yuqiong

**Affiliations:** Changchun Sci-Tech University, Faculty of Linguistic and Cultural Studies, Changchun 130600, China

## Abstract

With the continuous expansion of the Internet in China, network communication models and network services have become more and more complex, and with the increase of data types and diversification of data sources, network operation and maintenance projects have become more and more difficult. Passive statistical testing techniques for outliers are widely used, and many shortcomings have been pointed out, so there is an urgent need for improvement. After the research on the abnormal test of the text, it is determined that each method uses the visualization tool to simulate the data through the classification algorithm of the existing abnormal test and to identify the possibility of the data of each method and the PR diagram. The accuracy is counterintuitive. At present, Hallyu has a greater influence on the Internet, mainly in the fields of fashion and culture in Asian countries. Therefore, Korean language teaching has received widespread attention from the society, and combining cultural education with language teaching is an important way to improve the efficiency of language teaching. In the actual Korean language teaching work, a variety of Korean language materials are essential educational and teaching resources. The simulation results show that a large amount of training can make the DNN generate a better auto-encoder. In addition to strengthening the template for simulation training in deep learning, multiple supervisions of the data can be performed to reduce errors and improve efficiency.

## 1. Introduction

The scale of the network is constantly expanding and growing, the types of data and the range of users are also constantly expanding, and the demand for Internet abnormality checks is also increasing, which puts forward a relatively demanding index [1]. On the one hand, active performance detection technology uses dynamic identification of possible abnormal phenomena to quickly stop the location of fault points without the need to count traffic. This method can improve operating efficiency and reduce operating errors; on the other hand, in other words, based on network monitoring requirements, the performance indicators can be rationalized, and the range can be flexibly set [2]. Once the range is exceeded, the occurrence of outliers can be determined and rewards in time, which can increase the speed in each operation. If possible, it can reduce the user experience degradation caused by failures, improve the reputation of technology, increase the technology's market share, and avoid serious network failures caused by chain reactions [3]. When checking in this way, a reasonable acquisition adjustment process is very important, and the correct acquisition process will affect the important element of quality, and quality is the basis of overall operations. With the rapid development of the times and the continuous transformation of “Internet +” technology, it has surpassed the huge gap between scientific research and practical applications [4]. Many virtual scenes have gradually been integrated into actual scenes, enhanced human-computer interaction, and realized through artificial intelligence technology. A leapfrog breakthrough has achieved a new height of rapid development, making the speech recognition system more convenient and easy to use [5]. The purpose of in-depth learning is to strengthen the operation of the speech recognition system, improve the applicability of speech recognition technology in people's daily life, and meet people's higher requirements for speech recognition systems [6]. With the current acceleration of globalization, every country has constantly evolving. In recent years, Korean TV entertainment programs have developed rapidly. Due to the convenience of viewing the Internet, it has become a leader in spreading Korean culture, and the culture of China and South Korea has gradually merged. With the introduction and localization of some popular programs, the Hallyu craze is gradually heating up, and people's enthusiasm for Hallyu culture is increasing day by day. Under this circumstance, the text studies the background of structuralist semiotics, analyzes the willingness of Korean entertainment programs and typical cases, and summarizes the ideological supremacy thought from the back of the program. At the same time, we call on us to pay attention to the importance of spreading culture.

## 2. Related Work

The literature pointed out that Hawkins made a serious explanation in his 1980 paper, which is also the commonly used definition of abnormal testing today, and in the Hogg article on abnormal points in 1983, there is a genetic cause, which is a general algorithm [7]. Although collection and classification techniques are also widely used for anomaly detection, Knorr-Bremse's technique of describing outliers at a distance and using density to fit statistical definitions has been fully demonstrated [8]. According to data from the literature, voice recognition systems have been used in the home, and voice recognition technology, smart navigation, smart speakers, smart voice control, and auxiliary robots are also being used more and more. This fully proves the role of speech recognition technology in the rapid development of people. Therefore, if the in-depth study of the speech recognition system is strengthened, the speech recognition system can reach a higher level of service in human life, solve people's life problems, and, at the same time, make people's psychological life more enjoyable [9]. The literature pointed out that 2000 to 2010 was the golden period of rapid development of information technology, and speech recognition technology also carried out more in-depth research and exploration during this period. Researchers have also newly expanded the areas that the speech recognition system itself can contact, including noise signal processing, information recognition, speech line recognition, and intelligent speech synthesis [10]. The literature pointed out that when Li Keqiang proposed the “Internet +” action plan, the “Internet +” under the action plan quickly swept China and became a hot issue advocated by people. The so-called “Internet +” actually refers to “the combination of Internet innovation achievements and economic and social development to drive technological and social progress.” The emergence of the “Internet +” idea has had a huge impact and challenge on traditional university education [11]. Through the conflict and integration of quantum, a new type of education model called “Internet +” has been created. The literature points out that “Internet + education” shows that after breaking the relationship between active and passive and the subjective and passive relationship of existing Korean professors, they are organically combined to improve and optimize the relationship among professors, thereby achieving reversal of roles [12]. The “Internet + education” education model can better reveal the education ecology. By making the content of Korean learning more intuitive and vivid, and making students want to keep in touch with others, this is of great significance for cultivating students' active learning and creativity [13]. In the literature, at present, the Korean wave has had a greater impact on the fashion and cultural fields of Asian countries. Therefore, Korean language teaching has received widespread attention from the society, and combining cultural education with language teaching is an important way to improve the efficiency of language teaching [14]. Even in Korean classes, there is overlap between Korean and Chinese cultures, so it is necessary to actively introduce multicultural education programs, but many folk culture and historical understanding can also provide a good foundation for North Korean education through multicultural education. There are differences in some aspects. As Korean students, we will provide optimized Korean skills.

## 3. Research on Outlier Detection Model and Artificial Intelligence Language Feature Recognition

### 3.1. Research on the Outlier Detection Model

In a given data set, if we do not know whether the data itself are normal or abnormal, we always accept that most of the data are normal, so there is a quiet assumption that the concentration of nonmonitored data is always higher than normal. The situation is good.

We assume that the total amount of data is DT, the context data are GT, and the abnormal data are 0T.

(1) $$\begin{array}{c} G_{T}+O_{T}=D_{T|}|\frac{G_{T}}{O_{T}}\geq 1. \end{array}$$

Similarly, assuming that the data depend on a particular distribution, the number of outliers has different effects on statistics. Even in actual experiments, in order to measure whether an abnormal value is detected, it must be based on the Lubong attribute of the statistical data to be measured. For example, we suppose that the data come from a single variable.

Assuming that the average value of *X* + is 0, it is as follows:

(2) $$\begin{array}{c} \hat{E}=\frac{1}{N}\sum_{i=1}^{N}x_{i}. \end{array}$$

In order to discuss the minimum narrow variance matrix method, the method can start with the minimum volume and then reduce it under the premise of clustering the normal values. If the number of normal data is known as GT, the base of any number of GT is the smallest volume of an ellipse, in which only one point set including all normal values is generated. Assuming that the position coefficient is ∑ and the coefficient and ∑ are added together, the ellipse whose *σ* and radius length are defined by *Z* is as follows:

(3) $$\begin{array}{c} {\text{elli}}_{u,\Sigma }^{l}=\left\{x:{\left(x-u\right)}^{l}\Sigma^{-1}\left(x-u\right)<=l^{2}\right\}. \end{array}$$

The volume of the ellipse is as follows:

(4) $$\begin{array}{c} V\left({\text{elli}}_{u,\Sigma }^{l}\right)=vl^{d}\sqrt{\left|\Sigma \right|}, \end{array}$$

where *d* is the size, and *V* is the size in *d*.

(5) $$\begin{array}{c} v=\frac{\pi^{0.5\text{d}}}{\Gamma \left(0.5\text{d}+1\right)}. \end{array}$$

The radius *Z* is determined by the Mahalanobis distance, and the Mahalanobis distance is as follows:

(6) $$\begin{array}{c} \text{M dis}=\sqrt{{\left(x-u\right)}^{t}\Sigma^{-1}\left(x-u\right)}. \end{array}$$

Among them, *u* determines the location of the *X* collection point, and Σ determines the coordinate system. After obtaining the distance to the *N* data, we arrange them as 0 and remove the first Mahalanobis distance.

*l*_Gr_=M dis_*u*_^Gr^∑ includes the volume of GT standard data points as follows:

(7) $$\begin{array}{c} V\left({\text{elli}}_{u,\Sigma }^{l}\right)=vl_{G_{T}}^{d}\sqrt{\left|\Sigma \right|}. \end{array}$$

Denoted as *V*_Gr_, there are two ways to calculate the volume: let |∑| = 1; then, *V*_Gr_ depends on *l*_Gr_, and *l*_Gr_ depends on the parameters (*u*, ∑). Therefore, if the first Mahalanobis distance is measured as the smallest, the smallest volume can be obtained.

(8) $$\begin{array}{c} \left(u,\Sigma \right)=\underset{u,\Sigma 0}{\text{argmin}}\left\{l_{G_{T}}^{u,\Sigma }\right\}. \end{array}$$

Another way is to set *l*_Gr_ to 1.

(9) $$\begin{array}{c} u=\frac{1}{G_{T}}\sum_{i=1}^{G_{T}}x_{i},\\ \Sigma =\frac{1}{G_{T}}\sum_{i=1}^{G_{T}}\left(x_{i}-u\right){\left(x_{i}-u\right)}^{t}. \end{array}$$

Assuming that there are *G*_*T*_ in the normal point, it means that the function of *G*_*T*_ is the smallest volume. It is calculated that the experimental result when there is only one abnormal point has a large error, so the number of normal data can be determined.

(10) $$\begin{array}{c} G_{T}=f\left(V\right). \end{array}$$

When selecting *G*_*T*_ samples, with the increase in the total number of samples *N*, the choice of *G*_*T*_ is very large, and the amount of calculation increases rapidly. Therefore, in order to facilitate the calculation, we do not directly select *G*_*T*_, but proceed in the opposite direction, and gradually delete the data, and only the total amount of data is less than *N*/2. The specific steps are divided into three steps.

  Step 1: calculate the smallest ellipse that contains all the data
  Step 2: delete the abnormal point and record it once
  Step 3: repeat the first step, when the number of records reaches half, and do not repeat

The specific steps of the first step are as follows:

(1) Initial weight
  (11) $$\begin{array}{c} \omega_{i}=\frac{1}{N},\;i=1,\ldots ,N. \end{array}$$
(2) Calculate the position parameter *u* and the divergence parameter ∑
  (12) $$\begin{array}{c} u=\frac{1}{\sum_{i=1}^{N}\omega_{i}}\sum_{i=1}^{G_{T}}\omega_{i}x_{i},\\ \Sigma =\sum_{i=1}^{N}\omega_{i}\left(x_{i}-u\right){\left(x_{i}-u\right)}^{t}. \end{array}$$
(3) Calculate Mahalanobis distance and update weight
The expression of Mahalanobis distance is as follows:
  (13) $$\begin{array}{c} {\text{Mids}}_{t}=\sqrt{\left(x-u\right)\sum {\left(x-u\right)}^{t}}. \end{array}$$
If M dis_*i*_ > 1, we update the weight of the point:
  (14) $$\begin{array}{c} \omega_{i}=\omega_{i}\times \text{M }{\text{dis}}_{t}. \end{array}$$
(4) Judgment cycle

If the Mahalanobis distance of all points satisfies *Mdis* ≤ 1, we choose to terminate the operation, otherwise return to the first step. For the specific operation steps of the second step, see below equations.

Let *U*=(*x*_1_ − *u*,…,*x*_*N*_ − *u*)^*t*^, the covariance is as follows:

(15) $$\begin{array}{c} \text{Cov}=\frac{1}{U}UU{\;}^{\prime },\left|U_{-i}^{\prime }U_{-i}\right|\\ =\left(1-\alpha_{i}\right)\left|U{}^{\prime }U\right|, \end{array}$$

*u*_−*i*_ divided by *i* mean vector

(16) $$\begin{array}{c} \alpha_{i}={\left(U{\left(U^{t}U\right)}^{-1}U^{t}\right)}_{ii}. \end{array}$$

The larger the *a*_*i*_, the faster the ellipse becomes smaller after removing the *i*th sample. Determinant change graph is as shown in Figure 1, and ellipse change graph is as shown in Figure 2.

The analysis of Table 1 shows that although the accuracy of this method is 90%, it is very limited. One is that it is only applicable to single-modal data sets, and the other is that the result of whether the data are normal is also obvious.

The analysis of principal components is mainly used for dimension reduction. Under the premise of knowing sufficient information, reduce the dimensionality of data, reduce the amount of calculation, improve the display efficiency of experimental results, and remove abnormal points.

In the actual test, the solution of the principal component is mainly reflected in the two angles of maximum variance and minimum error, but the two are almost the same in nature, so we take the maximum variance as an example. As shown in Figure 3, data projection diagram, the retention of data information can be quickly obtained. It can be seen from this that there must be a suitable coordinate axis to make the data sufficiently discretized.

Data analysis shows that when the data are subtracted from the mean value, the image has no effect on the structure of the data, and only a rough translation transformation appears. Therefore, in a normal test, we usually de-average the data.

Therefore, if the data set is expressed as *X* =  {*x*_1_,…*x*_*n*_}, if the first main axis unit of the subject is *u*_1_, then the coordinate of each *x*_*i*_ under *u*_1_ is *x*_*i*_ · *u*, and the thought content of the principal component can be expressed as seeking new coordinates The sum of the distances between each point of the tie and the origin is the largest.

(17) $$\begin{array}{c} {\left\|Xu\right\|}^{2}=u{\;}^{\prime }X{\;}^{\prime }Xu, \end{array}$$

where ‖*u*‖ = 1, applying the Lagrangian multiplier method to obtain the following:

(18) $$\begin{array}{c} L\left(\lambda ,u\right)=u^{t}X^{t}Xu-\lambda \left(u^{t}u-1\right). \end{array}$$

We assume that the data are linearly related, so there must be changes in its structure: its main idea is to directly map all the retained data of the main axis to the original space, and the mapping point and the original point. The gap will reflect abnormal data.

Suppose the expression of the covariance matrix *C*_*X*_ of the data set *X* is

(19) $$\begin{array}{c} C_{x}=VDV^{t}. \end{array}$$

In this place, the contribution rate of the principal component needs to be used, and the number of retained feature vectors is determined by judging the contribution rate. We may wish to set the number of retained eigenvectors as *k* (*k* < *m*), and *V*_*k*_ is expressed as a matrix composed of all *k* eigenvectors. The data of the original data in the *V*_*k*_ matrix obtained in the experimental test is denoted as *X*_*K*_, and the expression of *X*_*K*_ is as follows:

(20) $$\begin{array}{c} X_{k}=XV_{k}. \end{array}$$

Pull back to the original space again to get the following equation:

(21) $$\begin{array}{c} X_{R}=X_{k}V_{k}^{t}. \end{array}$$

Define the weight of the *f*th eigenvector as follows:

(22) $$\begin{array}{c} \omega \left(i\right)=\frac{\sum_{i=1}^{t}\lambda_{l}}{\sum_{t=1}^{m}\lambda_{t}}. \end{array}$$

Therefore, we can express the scores of abnormal points in the following ways: method 1, use the contribution to set the lower limit to determine *X*_*R*_; method 2, make the feature vector gradually increase, and we can use the following formula to express the abnormal score of each data as follows:

(23) $$\begin{array}{c} s\left(x_{i}\right)=\sum_{l=1}^{m}\left(\left\|x_{i}-x_{R}^{l}E_{i}\right\|\times \omega \left(l\right)\right). \end{array}$$

The specific steps of the entire algorithm are as follows:

1. Obtain its eigenvalues and eigenvectors after computing the covariance matrix
2. Incrementally use the feature vector as the projection vector and pull it back to the original space
3. Calculate the abnormal point score to determine the degree of abnormality

#### 3.1.1. Experimental Results: By Confirming the Data, Adding Abnormal Points at Will, and Testing with the Above

Naive Bayes algorithm will have special subcontent for supervision, if all the labels of the data are known, and the data will be classified and reorganized with the help of probability, so that the new input data can quickly obtain its return content. The algorithm idea is simple, which is to make the conditional independence between the feature attributes, that is, *p*(*X*_*I*_, *i* = 1,…, *n*|*y*) = ∏_*i*=1_^*n*^*p*(*X*_*I*_*|y*), where *Y* is a categorical variable, and *Y* = 0, 1 in two categories.

The core formula of the whole algorithm is as follows:

(24) $$\begin{array}{c} p\left(y|x,i=1,\ldots ,n\right)=\frac{p\left(y\right)p\left(x_{i},i=1,\ldots ,n|y\right)}{\sum p\left(y\right)p\left(x_{i},i=1,\ldots ,n|y\right)}. \end{array}$$

#### 3.1.2. Outlier Discovery: Risk Scoring to Determine the Outlier

The simulation of the experimental test will generate pseudorandom numbers: one part is normal data, and the number is 200; the other part is abnormal data, and the number is 20. Let 150 and 15 be the training data.

The generated data set is the remaining data as shown in Figure 4.

In Figure 4, triangles indicate abnormal data, and circular data indicate normal data. Figure 4 can be obtained by data analysis, and the abnormal data in Figure 4 can be visually identified. The backtracking accuracy is up to 100%, but the decision-making accuracy is only 62.5% (see the backtracking curve). After the abnormal data are judged by the first 20% of the sample's risk score, the backtracking accuracy is full, so the first two samples are used as the judgment points. In the d-r curve, it can be seen that when the backtracking accuracy is exactly equal to 1, the decision-making accuracy decreases sharply, and the second inflection point is determined to be the optimal judgment point, and the values are exactly the same.

If the original training set and test set are directly put together and brought into the training model, the classification effect of Bayes will be displayed in a clearer way (see Table 2).

This model is generalized linear. It obtains the appropriate parameters through the maximum likelihood function under the same conditions, and then judges the category of the data according to the probability represented by each parameter.

This is a linear classifier. Set any one of *Y* = 0 or 1, the data are *X* = (*X*_1_,…, *X*_*n*_), and *X*_1_ is the n-dimensional data. The relationship between the probability of the classification label and the data can be expressed by the following expression:

(25) $$\begin{array}{c} p\left(y_{l}|x_{i}\right)=\frac{1}{1+e^{-\left(\beta_{0}+\beta_{N}x_{i}\right)}},\\ \beta_{N}=\left(\beta_{1},\ldots ,\beta_{n}\right). \end{array}$$

Finally, the parameters and goodness of fit obtained from the model need to be tested. For the test of each parameter, the commonly used statistic is the Wald test, and the goodness of model fit is often judged by the Akaike information criterion.

*π* (*y*_*i*_) is the risk score when abnormal, and the real data are determined by the d-r curve, as shown in Table 3.

The AIC value was 44.081, and the overall model passed the test. The semisupervised anomaly detection and analysis method is only suitable for the labeled data in the data set. Because there are less data that match, we can only slowly explore the rules and use semisupervised anomaly detection and analysis to determine the authenticity.

The simulation example mainly uses the semisupervised detection method to actually use the time series data generated by simulation. In order to better realize the simulation example, we add abnormal points to test and outlier detection result of simulated sequence as shown in Table 4. The difference between the estimated value of the simulation parameter and the real value is shown in Table 5.

From the abnormal point detection results of the simulation sequence in Table 4 and the difference between the estimated value of the simulation parameter and the real value, we can find that we can identify all the abnormal point data, and the estimated value and the actual value of the model parameter are more similar.

After the above simulation, a sequence of 1200 length will be generated, and the last 200 data will be selected for analysis. In this batch of data (200), we set 3 additional anomalous points, and set them at positions 40, 90, and 120, respectively. The anomalous effect sizes are 6, 5, and 5, respectively. The final data of the time series diagram of the simulation sequence are shown in Figure 5.

The outlier detection result is shown in Table 6.

As can be seen from the above table, the type and location are the abnormal points. MA model abnormal point detection is shown in Figure 6.

The method of stationarity test is similar to the above model, so I will not repeat it. Here, it is a brief introduction to the process of ARMA model identification and order determination.

It can be seen from the EACF information of the simulation sequence in Figure 7 that the (1, 1) model should be used to detect abnormal points. Outlier detection result of simulated sequence is shown in Table 7.

### 3.2. Research on Artificial Intelligence Speech Feature Recognition

Language recognition technology: Convert human speech into machine language. The process of its random model method: speech signal preprocessing-feature extraction-first classification in the speech model library and then matching-language processing in the language model library-so that the computer can recognize. With the progress of the times, further breakthroughs are still needed in the study of speech recognition systems. Although speech recognition technology has also achieved human-machine communication, the machine is always a machine, and the language model for dictation recognition needs to be improved. There is no grammatical model based on linguistics for recognition and understanding. At the same time, there is still need for improvement in noise processing and multilanguage hybrid recognition. Therefore, speech recognition technology still needs to be further improved.

Traditional speech recognition relies on manual extraction of features to generate acoustic models and speech models. These two models are still too restrictive and will definitely be affected by human factors. Deep neural network can perform automatic feature extraction, so the auto-encoder generated by DNN is used to accurately extract features, and then truly realize human-computer interaction.

Feature extraction is to find features that can represent the province of the voice signal from a large amount of information carried by the voice signal. Due to the unique and diverse characteristics of the actual environment, deep learning has a big advantage. It can generate an auto-encoder to enable the neural network to provide a better model so that the neural network model can reduce unnecessary judgments during training and obtain the optimal solution. A lot of training can make DNN generate better auto-encoder. In addition to strengthening the simulation training template in deep learning, multiple supervision of data can also be performed to reduce errors and improve efficiency.

With the progress of the times, people hope to have emotional conversations with artificial intelligence, turning it into a combination of “partners” and “servers.” Therefore, the technical problems of speech emotion recognition are urgently needed to be solved and integrated into facial expressions and speech organ movement data, which will help artificial intelligence to obtain emotion recognition. The future speech recognition system may provide people with a combination of “partners” and “servers” through deep learning so that they can recognize the emotions of each person being served.

## 4. Research on the Spread of Korean Language and Culture

### 4.1. Problems in the Spread of Korean Language and Culture

Driven by the background of the times, the “Internet + education” model has gradually become mature, allowing the outdated traditional education system to be reshaped, and a large number of high-quality learning resources and educational resources have been improved, and the educational content, methods, and approaches have been improved. In this way, education resources that originally only exist in developed areas can be popularized throughout the country, and children in some relatively backward and remote areas and other areas with relatively poor education resources can also get better quality education. This is to a large extent that the above solves the problem of irrational distribution of education resources in China, and allows education to develop fairly. However, while enjoying the advantages of “Internet+” in educational development, we must also clearly recognize the challenges we face. Under this educational model, there are still certain problems in Korean teaching in colleges and universities, which are mainly manifested in the following aspects.

After the “Internet +” education was put forward, the state paid more attention to this new education model and proposed relevant support policies. With the support of policies, the current education model has been developed toward an informatization model, and the software and hardware conditions in the student education environment have been greatly upgraded. Despite the support of such policies, some colleges and universities still have insufficient investment in education funds, and the degree of informatization of hardware resources has not been fully popularized. The hardware resources are relatively outdated. Some areas were even in the original mode and still used. Traditional teaching methods do not use the Internet or multimedia, and their degree of informatization lags far behind developed regions. Although the “Internet +” era has allowed rapid development in some fields, due to the limitations of certain hardware devices, the teaching efficiency of Korean language classrooms in colleges and universities has been slow to improve. Therefore, the hardware environment of education informatization still needs to be improved, which is also one of the problems that the country urgently needs to improve in the reform of student education.

Weak emotional guidance is the main problem faced in the context of “Internet + education.” In the vast ocean of Internet knowledge, the knowledge contained in it is integrated and combined, and it is also characterized by rich resources and a variety of styles. This directly leads to restrictions on the learning caliber of college students, although a wide range of knowledge can be greatly improved. The students' autonomous learning ability, however, makes the connection between teachers and students increasingly weak. If things go on like this, the emotional communication between teachers and students will gradually be weakened. The status of teachers is weaker than multimedia and gradually tends to be marginalized. In addition, for some college students with poor foundations, how to find the knowledge of the Korean language they need in the vast ocean of study is also a major problem they face. If the above two situations continue to progress, if relevant measures are not used to contain them, the strong will become stronger and the weak will become weaker.

### 4.2. Suggestions for the Spread of Korean Language and Culture

At present, the Korean language teachers in Chinese universities have less theoretical knowledge and practical operations in Korean cultural communication. Therefore, Korean teachers in universities can conduct activities such as outbound travel and overseas training to improve their cultural literacy. In addition, we can also hold various salon exchange meetings with foreign teachers, foreign students, and returned teachers in our school to indirectly understand the real Korean culture, thereby increasing our cultural literacy in Korean.

When students study language subjects, they will definitely use communication to strengthen their own learning achievements, and learning Korean is no exception. Therefore, an important indicator of Korean teaching is to enable students to use Korean for stable and convenient communication. Therefore, teachers should actively build an efficient and convenient communication platform for students. Let real communication strengthen students' Korean foundation and application skills. Therefore, a high-quality communication platform can enable students to carry out actual communication, which can promote students to improve the foundation, learning ability, and application ability of the Korean language, and at the same time strengthen the students' Korean cultural literacy. Culture is a kind of spiritual wealth. In the work of Korean cultural education, teachers need to guide students to appreciate the knowledge of Korean history, politics, and economy, so as to enhance students' interest in Korean culture and strengthen students' cultural literacy.

The Chinese and Korean cultures are harmonious but different. Teachers will have different opinions on using Chinese culture and Korean culture to understand some Korean idioms and proverbs. For this kind of teaching work, it is necessary to compare the historical backgrounds and customary expressions of the two countries with examples, so as to guide students to understand more accurately. At the same time, due to the integration of cultures of various countries, China has also introduced many Korean videos and Korean songs, which can improve the Korean cultural literacy of students and help students understand Korean culture. Teachers need to combine normal teaching content with rich Korean cases in their teaching work, and compare the cultural and language characteristics of China and South Korea with examples, so as to improve students' Korean comprehension.

In the actual Korean teaching work, a variety of Korean materials are indispensable educational and teaching resources. At the same time, because modern Korean materials are presented in fashion video works and song works, and teachers' correct quotations in education and teaching work can improve students' learning enthusiasm to a certain extent. Moreover, a correct case analysis of materials will inevitably enhance students' understanding of Korean expressions, improve students' ability to analyze Korean film and television works, and further enhance students' interest in learning Korean culture, thereby further improving students' Korean cultural literacy and the understanding and use of Korean.

## 5. Conclusion

This article first summarizes the common algorithms required for experimental testing, and then divides the used algorithms into two types of algorithms with unsupervised features according to whether the data selected in the experiment have labels, so as to use algorithm cases for practice and analysis. The introduction of unbalanced abnormal experimental data in the actual experimental process leads to small fluctuations in the accuracy of the prediction of the normal point, making the result incompletely accurate. And because the foundation of the model is backtracking accuracy and decision-making accuracy, the quality of the model is also determined by the data's backtracking accuracy and decision-making accuracy. In addition, the ROC diagram is used to directly observe the quality of the model. The more the ROC curve of the model deviates from the upper left corner, the worse the model is, and vice versa. According to the algorithm summary of the selected algorithm, we accurately combined Dirichlet and OCSVM to discover and study abnormal points. OCSVM can mine the abnormal points in the data of all patterns, while Dirichlet can judge and analyze the patterns of the data. This method belongs to the unsupervised type, but its performance is better than the supervised algorithm logistics. In the following article, we first introduce the research background of speech emotion recognition, point out various problems in the field of speech emotion recognition, and introduce in detail the current research status of speech emotion recognition at home and abroad and the significance of studying speech emotion recognition. In terms of model selection, we first introduced the working principle of ANNs and introduced its model for speech recognition. In order to more effectively mine the information in the features, we also introduced some excellent characteristics of combining a variety of different neural networks for speech recognition emotion technology.

This project requires the cooperation, cooperation, and mutual restriction of personnel at all levels to form an organic development prospect, thereby building a national image system. Generally speaking, the external dissemination of national image culture needs to be realized in a systematic way of thinking in order to show a good national face to the outside world. In view of the above research, “Internet +” welcomes the high enthusiasm for the entire era, making every industry in it usher in development opportunities. Among them, artificial intelligence speech recognition technology also brings huge opportunities to Korean classrooms in colleges and universities. While the development of education is enjoying the dividends of the Internet era, it must continue to discover and eradicate defects, and constantly break through technical difficulties. All in all, in the context of the “Internet+” era, Korean classrooms in colleges and universities must seize the opportunity and make full use of teaching resources and teaching advantages to build a new Korean teaching system and realize the reform of Korean teaching in colleges and universities.

## Figures and Tables

**Figure 1:** Determinant change graph.

**Figure 2:** Ellipse change graph.

**Figure 3:** Data projection.

**Figure 4:** Naive Bayes simulation data.

**Figure 5:** Time series plot of simulation sequence.

**Figure 6:** MA model abnormal point detection.

**Figure 7:** EACF information for the simulation sequence.

**Table 1:** Judgment accuracy.

(Total sample size, abnormal points)	(50, 10)	(100, 10)	(200, 10)	(200, 20)	(300, 20)
*D*	0.91	1	1	1	1
*r*	1	1	1	0.95	0.9

**Table 2:** Confusion matrix for Bayes classification.

Columns represent real data	Positive	Negative class
Positive	0.95	0.05
Negative or unknown	0.02	0.98

**Table 3:** Significance test table.

Intercept *c* = −7.9499		*β*_1_ = 0.8064	*β*_2_ = 0.8394
*p* value	≤0.01	0.003	0.001

**Table 4:** Outlier detection result of simulated sequence.

Types of outliers	Location of outliers	Size of abnormal effect	Actual setting exception size
AO	40	5.024	6
AO	90	3.741	5
AO	150	5.817	5

**Table 5:** The difference between the estimated value of the simulation parameter and the real value.

Model parameters	Estimated value	Actual value
*φ*1	0.9055	1
*φ*2	−0.4082	−0.5
Intercept term	−0.1031	0

**Table 6:** Abnormal point detection results of MA model.

Types of outliers	Location of outliers	Size of abnormal effect	Actual setting exception size
AO	40	6.115	6
AO	90	5.411	5
AO	120	4.713	5

**Table 7:** Outlier detection result of simulated sequence.

Types of outliers	Location of outliers	Size of abnormal effect	Actual setting exception size
AO	40	−5.428	−5
AO	90	4.733	5.5
AO	120	5.095	5

## Data Availability

The data used to support the findings of this study are available from the author upon request.
